This article has been retracted.

# Genetic regulation of salt stress tolerance revealed by RNA-Seq in cotton diploid wild species, *Gossypium davidsonii*

**DOI:** 10.1038/srep20582

**Published:** 2016-02-03

**Authors:** Feng Zhang, Guozhong Zhu, Lei Du, Xiaoguang Shang, Chaoze Cheng, Bing Yang, Yan Hu, Caiping Cai, Wangzhen Guo

**Affiliations:** 1 State Key Laboratory of Crop Genetics & Germplasm Enhancement, Hybrid Cotton R & D Engineering Research Center, Ministry of Education, Nanjing Agricultural University, Nanjing 210095, China; 2 Yunnan Ice Harbor Biotechnology Co. Ltd, Kunming 650000, China

## Abstract

Cotton is an economically important crop throughout the world, and is a pioneer crop in salt stress tolerance research. Investigation of the genetic regulation of salinity tolerance will provide information for salt stress-resistant breeding. Here, we employed next-generation RNA-Seq technology to elucidate the salt-tolerant mechanisms in cotton using the diploid cotton species *Gossypium davidsonii* which has superior stress tolerance. A total of 4744 and 5337 differentially expressed genes (DEGs) were found to be involved in salt stress tolerance in roots and leaves, respectively. Gene function annotation elucidated salt overly sensitive (SOS) and reactive oxygen species (ROS) signaling pathways. Furthermore, we found that photosynthesis pathways and metabolism play important roles in ion homeostasis and oxidation balance. Moreover, our studies revealed that alternative splicing also contributes to salt-stress responses at the posttranscriptional level, implying its functional role in response to salinity stress. This study not only provides a valuable resource for understanding the genetic control of salt stress in cotton, but also lays a substantial foundation for the genetic improvement of crop resistance to salt stress.

Plants face a multitude of biotic and abiotic stresses during their lifespan. Salt stress is the most serious threat to agriculture and to the environment in many parts of the world. Salinity impairs cellular osmotic and ionic homeostasis and also compromises photosynthesis, depletes cellular energy, and leads to redox imbalances. As a consequence, inhibition of photosynthesis, metabolic dysfunction, and damage to cellular structures lead to abnormal growth and even death^1^.

Plants exhibit a variety of responses to salt stress that enable them to tolerate adverse conditions involving physiological, biochemical, and molecular processes. Generally, the molecular mechanisms are relatively complex compared to the physiological and biochemical process. Although more work needs to be done to elucidate these molecular mechanisms, an increasing number of studies have focused on this field and have achieved a consensus in model plants such as *Arabidopsis* and rice^2^. The studies have shown that receptors in the plasma membrane transfer stress information to the cell body when salt stress is perceived. Then stress-activated transcription factors initiate transcriptional reprogramming by signaling transmission that finally results in changes at the protein level. Eventually, de novo-synthesized structural or enzymatically active proteins directly or indirectly participate in the maintenance of osmotic, ion, and redox balance^3^,^4^. It is clear that signaling pathways play a pivotal role in this process, including various hormones, salt overly sensitive (SOS), mitogen-activated protein kinase (MAPK) cascade and reactive oxygen species (ROS) signaling pathways^5^,^6^. Extensive studies have found that these signaling pathways are not acting individually, but coordinate their actions to enhance tolerance to salt stress^6^,^7^. In addition, alternative splicing, miRNA and chromatin modifications, and epigenetics also contribute to salt tolerance^8^,^9^,^10^.

Although cotton is a relatively salt-tolerant species, the growth and development of this plant can still be greatly affected by adverse salt conditions. As such, researchers have focused on investigating the key molecular factors involved in the response to salt stress, and have attempted to breed salt-tolerant cotton cultivars. Transcription factors are considered the most important regulators of gene expression. In cotton, the roles of transcription factors such as *WRKY*, *CCCH-*type zinc finger, *NAC*, *ERF*, and *DREB*, in salt tolerance have been well documented. Evidence from transgenic plants has demonstrated that *GhWRKY39-1* and *GhDREB1* genes could function as positive regulators to enhance abiotic stress tolerance^11^,^12^. In addition, over-expression of the rice NAC gene, *SNAC1*, could also improve salt tolerance in transgenic cotton^13^. Key regulators in the salt stress response are often involved in signal transduction pathways and protein kinase is the most typical player at this level. *GhMKK1*, *GhMKK4*, and *GhMPK2* positively regulate salt tolerance in different pathways^14^,^15^,^16^, whereas cotton *GhMPK6a* negatively regulates osmotic tolerance and *GhMKK5* reduces the tolerance to salt and drought stress in transgenic *Nicotiana benthamiana*^17^,^18^. Previous studies have shown that cotton CBL-interacting protein kinase gene (*GhCIPK6*) and SnRK2 are also involved in abiotic stress tolerance^19^,^20^. The involvement of ion transport in the salt stress response has also been exhibited. Ectopic expression of the H^+^-PPase gene from *Thellungiella halophila* resulted in higher salt tolerance in transgenic cotton^21^. The Na^+^/H^+^ antiporter plays an important role in salt stress, and over-expressing *AtNHX1* in cotton can improve salt tolerance^22^. In addition, *GhSOD1*, *GhCAT1*, and *GhMT3a*, which act as ROS scavengers, participate in the salt stress response in cotton^23^,^24^. Over-expression of the cotton annexin gene, *GhAnn1*, confers tolerance to salt stress of transgenic plants^25^.

Although a number of cotton genes have been shown to participate in salt stress, most have been studied by ectopic expression. Furthermore, few studies have focused on the regulatory networks in cotton. Hence, the links between these players in the response to salt stress in cotton are difficult to define. Transcriptomic analysis provides detailed information about gene expression at the mRNA level and is widely used to screen candidate genes involved in stress responses. Recent transcriptomic studies have contributed to our knowledge of the molecular regulatory pathways to salt stress tolerance and adaptation in cotton, with several genes and miRNAs identified to play important roles in the response to salt stress^26^. However, their mechanisms are not well known because the studies focused on the early transcriptional changes in response to salt stress, or on their activity in either leaves or roots rather than in both. In fact, roots, the first tissue to perceive salt stress, and leaves, the organ central in the control of water loss, play fundamental roles in salt stress^27^.

Here, we aimed to identify the key genes involved in responses to salinity stress and their crosstalk, using RNA-Seq analysis in the roots and leaves of *G. davidsonii*, a cotton D-genome diploid species with important properties of salinity stress resistance. The stress-tolerance properties of *G. davidsonii* were first confirmed by detecting the various reported physiological indexes related to salt tolerance^28^. Then, the cotton transcriptomes from salt-treated and well-watered roots and leaves were compared. Ultimately, the influence of crosstalk between the key genes on gene expression and cellular and physiological responses to enable adaptation and/or resistance to salt stress were investigated. This study not only provides new avenues to test existing research hypotheses but also helps to shape new ideas that could form a solid foundation for effective engineering strategies to increase salt stress tolerance in cotton.

## Results

### Phenotypic and physiological responses to salt stress in *G. davidsonii*

The salt tolerance properties of *G. davidsonii* were first observed by comparing this species with two other *G. hirsutum* accessions, ZS9612 and Z9807, which exhibited sensitivities and insensitivities to salinity stress, respectively. We found that *G. davidsonii* showed a higher relative photosynthetic rate (Fig. 1a) and relative leaf water content after salt stress (Fig. S1) than ZS9612, although these values were much lower in both genotypes after 12 h of exposure to NaCl compared with controls (data not shown). Furthermore, the Na^+^/K^+^ ratio was significantly lower in *G. davidsonii* (Fig. 1b,f), suggesting that Na^+^/K^+^ homeostasis is more balanced in *G. davidsonii* compared to ZS9612. Moreover, *G. davidsonii* exhibited lower lipid peroxidation (Fig. 1d,h), more superoxide dismutase (SOD), active antioxidant enzymes (Fig. 1c,g), and higher proline accumulation (Fig. 1e,i) than ZS9612. Importantly, the physiological indexes measured in *G. davidsonii* showed similar or better tolerance characteristics than that in the salinity insensitive accession Z9807 after salt stress (Fig. 1a–i). Taken together, *G. davidsonii* possesses important properties of salt tolerance.

### Processing and mapping of Illumina reads

Using diploid D-genome species *G. davidsonii*, RNA-Seq analyses were performed on two independent biological replicates of each sample in this study. RNA samples were collected from both the roots and leaves at 12 h, 24 h, 48 h, 96 h, and 144 h post salt stress (200 mM NaCl). *G. davidsonii* seedlings grown in normal conditions were used as controls. In total, 40 separate libraries were generated. The reads generated by the Illumina Hiseq2000 were initially processed to remove adapter sequences and low-quality bases. The reads were then mapped to the sequenced *G. raimondii* genome using Tophat^29^, which allows the identification of splicing events involving novel exons and novel intergenic transcripts. Approximately 1.61 billion valid reads, each 101 nucleotides long, and roughly 162.6 Gb of nucleotides were obtained. On average, 40.25 million clean reads were obtained from each library, and 59.74–84.47% of the total reads were aligned to the reference genome. The aligned sequences were assembled with Cufflinks guided by a reference annotation from JGI Genomes (*G. raimondii* 2.0). The reads mapping to the genome are shown in Table S1 and the workflow of RNA-Seq analysis in Fig. 2. The RNA-Seq assays revealed that there were a total of 157,953 transcripts and 43,219 unigenes with 85.71% (37,046 unigenes) annotated genes and 14.29% (6245 unigenes) novel genes (Table 1).

### Differentially expressed gene identification in leaves and roots under salt stress and normal conditions

From each biological replicate, the transcript abundance of each gene was estimated by fragments per kilobase of exon per million fragments mapped (FPKM). Cufflinks^30^ was used to calculate the differential expression pattern. A cutoff q value ≤ 0.05 and fold change ≥ 1 was used for identifying differentially expressed genes (DEGs). Integrating the reproducibility between the biological replicates, we totally found 4,744 DEGs in roots and 5,337 in leaves following the salt treatment. The distribution of these genes is shown in a Venn diagram (Fig. 3A), which highlights that 1,837 DEGs were commonly identified in the two tissue types. Interestingly, there were several more DEGs in the leaves than in the roots, implying that the leaves undergo more complicated transcript regulation after salt treatment. More genes were up-regulated than down-regulated in both roots and leaves in response to the salt stress (Fig. S2). In roots, approximately 70% of the total DEGs were identified at 12 h and 24 h post stress and far fewer DEGs were found at 48 h, 96 h, and 144 h post stress. However, in leaves, most of the DGEs were identified after 24 h post stress (Fig. 3B). These results imply that the expression pattern in roots changed rapidly after salinity stress, while the leaves responded to the stress after 24 hours. It was shown that 51 genes were differentially expressed in all root samples comparisons and 67 in all leaf comparisons (Fig. 3C,D). The expression of these genes showed either a continuous up-regulation pattern or a continuous down-regulation pattern. Only two of the DEGs (*Gorai.004G128700*, which encodes a UDP-Glycosyltransferase superfamily protein, and *Gorai.002G222900,* which encodes alcohol dehydrogenase 1) were up-regulated at all salt-stressed stages in both tissues (Fig. 4). Alcohol dehydrogenase (ADH) is an important zinc-containing enzyme in plants, which plays a crucial role in stress responses to drought, cold, and invasion by biological pathogens^31^,^32^. The function of UDP-Glycosyltransferase under salt stress is unclear, but several previous studies indicate UDP-Glycosyltransferase is related to salt stress^33^,^34^.

### GO enrichment analysis of the DEGs

To understand their function, we mapped all of the DEGs to terms in the GO database using agirGO^35^. GO category enrichment analysis was performed using P-value of 0.05 adjusted by false discovery rate (FDR) as the cutoff. In our expression data, 2,304 (43.2%) and 1,896 (40.0%) of DEGs in leaves and roots, respectively, were annotated. ‘Response to stimulus’ (GO:0050896) was the most significantly enriched GO term both in leaves and roots (Fig. 5). GO enrichment analysis revealed an enrichment of genes involved in plant responses to chemical stimuli, organic substances, abiotic stimuli, reactive oxygen species, osmotic stress, and salt, as well to hormone stimuli both in leaves and roots. More GO terms related to ‘response to stimulus’ were identified in roots (Fig. 6) than that in leaves (Fig. 7), implying that a more complicated physiological process occurred in roots than that in leaves when the plant was stressed by salinity. Furthermore, in order to understand the dynamic expression patterns of DEGs under salt stress, several key terms were investigated (Table S2). It revealed that “response to stress” and “ion transport” genes reached a higher expression level at early stages in roots but at late stages in leaves. Moreover, according to the number of DEGs in the categories of “inorganic anion transport” and “monovalent inorganic cation transport”, ion stress was not significant at early stages in leaves, whereas osmosis stress had been perceived at these stages. This result is consistent with previous study which showed that plants are initially affected by osmotic stress then subjected to ion stress^36^. In addition, GO category analysis was also performed for common DEGs in both tissues. The functions of 51 common DEGs in roots were mainly “transport”, “response to stimulus”, and “membrane part”, and 67 common DEGs in leaves were mainly involved in “metabolic process”, “regulation of development process”, “response to stimulus” and “hydrolase activity”.

### DEGs involved in key biological process

Based on function annotation, these DEGs were allocated into several biological processes, involved in hormone metabolism, mitogen-activated protein kinase (MAPK) cascade and Ca^2+^-related kinase regulation, ion homeostasis, photosynthesis process, ROS production and scavenging, and transcription factor regulation. It has been established that hormones, MAPK cascades, and Ca^2+^ signaling pathways play important roles in responses to salt stress in *Arabidopsis* and rice^6^. However, many of the main factors in these signaling pathways have yet to be determined. In our study, the key regulators of hormones were consistent with previous reports, especially for abscisic acid (ABA), jasmonic acid (JA), and ethylene (ET) (Fig. S3a). For example, it has been demonstrated that *NCED3*, *PYR/PYL/RCARs*, *SnRK2s*, *AtMYB20*, and *PP2C* played an important role in plant salt stress via ABA mediated pathways^37^,^38^,^39^,^40^. In the present study, *NCED* and *PP2C* genes were dramatically up-regulated while almost all *PYR/PYL/RCARs* were down-regulated (Fig. S3a). In addition, DEGs coding for some key factors in MAPK cascades and Ca^2+^ signaling pathways in response to salt stress were also found (Fig. S3b), and these agreed with those described in previous reports^41^,^42^. Further, we focused on mining the DEGs linked to signaling pathways, metabolism, and developmental processes that have been previously neglected in cotton.

### DEGs involved in ion homeostasis

Maintaining ion homeostasis by ion uptake and compartmentalization is crucial for normal plant growth during salt stress. At the cellular level, the Salt Overly Sensitive (SOS) signaling pathway has been well documented^38^. In our study, SOS3 (myristoylated calcium-binding), SOS2 (serine/threonine protein kinase; a member of the SnRK3 family), and SOS1 (a Na^+^/H^+^ antiporter), which are basic components of the SOS signaling pathway, were investigated. As expected, SOS2 transcription was upregulated in roots and leaves, and SOS1 was up-regulated in leaves at 144 h after exposure to salt stress. The level of SOS3 transcription was unchanged, while SOS3-like calcium binding protein 8 (also known as calcineurin B-like CBL10) was up-regulated in roots at 12 h and 24 h after salt stress (Fig. S3c). As an alternative regulator of SOS2, SCaBP8 is more prominent in roots in *Arabidopsis* than SOS3^43^. Therefore, we speculated that the functions of SOS3 and *SCaBP8* in the SOS signaling pathway may have interspecific differences.

Furthermore, the vacuolar sequestration of Na^+^ via the *NHX2* tonoplast antiporter is also important in Na^+^ homeostasis at a cellular level. In our study, *NHX2* (*Gorai.008G008200*, *Gorai.007G264500*, and *Gorai.005G057100*) was found to be up-regulated in both root and leaf tissues (Fig. S3c). Moreover, the maintenance of high intracellular K^+^/Na^+^ ratios is important to avoid Na^+^ poisoning. Several genes involved in this process were found to be up-regulated, including *HKT* transporters, the potassium transporters *KUP1* (*Gorai.011G051700*), *KUP2* (*Gorai.009G292800*), and *KUP11* (*Gorai.005G267900* and *Gorai.008G049100*), and a shaker-type potassium channel gene, *SKOR* (*Gorai.009G114200*). In addition, three plasma membrane *ATPase* genes involved in ion homeostasis were also up-regulated in both tissues (Fig. S3c).

### DEGs involved in photosynthesis

Significantly, salinity impairs cellular ionic, osmotic homeostasis and redox balance but additionally compromises photosynthesis. However, as a leaf-specific biological process, the mechanism of this has not been widely investigated. In our study, through GO analysis, we found that “photosynthesis, light reaction” (p = 9.9e-13) and “photosynthesis” (p = 2.3e-12) were significantly enriched in leaves under salt stress. 123 DEGs were obtained from the GO term “photosynthesis”. Pathway analysis by mapman (Table S3) revealed that various components of photosynthesis were down-regulated from 96 h after salt stress in leaves, which was followed by ion stress and osmotic stress. Further analysis showed that these down-regulated genes were mainly involved in the light reaction, including *LHC* (18) (a type of photosynthetic pigments-related genes), *PSB* (33) (a component of photosystem II), *PEI* (6) (a component of cytochrome b6), *PSA* (24) (a component of photosystem I), and several genes related to ATP synthase (9) (Fig. S3d). In addition, eight *RuBisCO* subunits were found to be down-regulated (Fig. S3d). *RuBisCO* is a key enzyme in the first step of carbon fixation in the Calvin cycle^44^.

### DEGs involved in ROS production and scavenging

In response to salt stress, ROS accumulation depends on the balance between ROS production and scavenging^45^. In the study, the H_2_O_2_-producing genes, *RBOHs* (respiratory burst oxidase homologs), were significantly up-regulated in both root and leaf tissues when suffering salt stress (Table S4, Fig. S3e). Simultaneously, ROS scavenging systems were markedly influenced, showing different expression patterns under salt treatment. 14 and 11 members of ascorbate peroxidase (POD) family, one of the three major families of ROS detoxifying enzymes, were up-regulated in roots and leaves, respectively. However, only two and one catalase (CAT) genes were up-regulated in roots and leaves, respectively, and no change was found in superoxide dismutase (SOD) expression. In addition, the transcript level of genes related to antioxidant metabolites, such as glutathione and tocopherols, were also changed. Moreover, genes coding for peroxiredoxins (PRXs) and glutaredoxins (GRXs) showed completely opposite expression patterns in leaves. Two PRX genes were totally inhibited, whereas two GRX genes were up-regulated. Meanwhile, most of the glutathione S-transferase (GST) genes were significantly up-regulated both in roots and leaves at different times after salt stress (Fig. S3e). These results suggest that the enzymatic pathways of POD, GST, and CAT gene families primarily function in protecting cotton against oxidative damage under salt stress.

### DEGs involved in transcription factors

Numerous studies have demonstrated the important roles of transcription factors in plant defenses against abiotic stresses in a variety of species^46^,^47^. In our study, GO analysis showed that transcription regulator activity was significantly enriched in *G. davidsonii*. 618 and 611 DEGs were identified in roots and leaves, respectively. These TFs were classified into 57 families, with 1 group of unclassified factors. In addition, salt-stress markedly affects several super-families of TFs, including *AP2/EREBP*, *bZIP*, *bHLH*, *MYB*, *NAC*, and *WRKY*. In roots, most TFs were regulated at 12 h and 24 h after salt stress (Fig. S4). However, in leaves, most TFs were significantly differentially expressed at 96 h and 144 h after salt stress (Fig. S4). Interestingly, some tissue-specific regulated TFs were found to be altered in our data; i.e. three plant-specific transcription factor *YABBY* family proteins (*Gorai.002G160300, Gorai.005G262300*, and *Gorai.013G021300*) were exclusively regulated in leaves. Their expression pattern is different, for instance, *Gorai.002G160300* was up-regulated only at 48 h, *Gorai.005G262300* was up-regulated only at 96 h, but *Gorai.013G021300* was down-regulated only at 96 h. The TF families which contained greater than 10 members are shown in Fig. S4.

### Salt stress induces genome-wide alternative splicing in *G. davidsonii*

Alternative splicing can enhance transcriptome plasticity and proteome diversity. In plants, alternative splicing can manifest at different developmental stages, and is frequently associated with specific tissue types or environmental conditions such as abiotic stress^48^. After application of the strict filter, we identified 14,172 alternative splicing events in 6,798 genes composed of two or more exons, with an average of 2.08 alternative splicing (AS) events per gene. Of them, four main alternative splicing categories (Fig. 8a): intron retention (IR), exon skipping (ES), alternative acceptor site (AA), and alternative donor site (AD), involving 85.5% alternative splicing events, were further analyzed. We found that IR accounted for 35.73% of all AS events and it was the most abundant AS pattern, followed by AA (29.25%), AD (12.76%), and ES (7.71%) (Table S5). This is consistent with that IR is the major splicing pattern in *Arabidopsis*^49^. Moreover, no matter in roots or leaves, more novel AS isoforms were generated under salt stress condition when compared with normal condition and some AS events were tissue-specific (Fig. S5). Gene annotation implied that a multitude of genes that play core roles in the response to abiotic stress were involved in alternative splicing events, such as *MAPK*, *bHLH* and zinc finger transcription factors, cytochrome P450 and so on. Further, four main AS patterns and mutually exclusive exon (MEE) pattern was selected randomly and verified by RT-PCR and qRT-PCR (Fig. 8b–f). The results indicate the presence and spatio-temporal regulation of alternative gene splicing under salt stress conditions in cotton.

### Validation of the RNA-Seq data by real-time qRT-PCR

In order to prove the reliability of the RNA-Seq data, real-time qRT-PCR was performed on the same RNA pools that had been previously used for the next-generation sequencing. 30 genes, including 10 up-regulated, 10 unchanged, and 10 down-regulated genes, were randomly selected for qRT-PCR analysis. To corroborate the expression levels measured by RNA-Seq, the ratio of expression levels between salt stressed tissues and controls using RNA-Seq was compared to the ratio of expression as measured by qRT-PCR. The qRT-PCR results were significantly correlated to the RNA-Seq data in both leaves and roots (R^2^ = 0.863 and 0.886, respectively) (Fig. 9). The validation experiments support the reliability of the relative values provided by the RNA-Seq analysis.

## Discussion

Salinity is a prevalent abiotic stress that limits cotton growth and development in the form of osmotic stress, which is then followed by ion toxicity. To date, the salt tolerance mechanism in cotton has been less studied. Although roots and leaves are two of the most important tissues in the response to salt stress, most previous studies have only focused on one of these tissues. The cotton diploid species, *G. davidsonii*, shows important properties of salt stress tolerance (Fig. 1). In this study, the roots and leaves of *G. davidsonii* seedlings exposed to salt stress were used for RNA-Seq analysis. Thus, this may further elucidate the complex mechanisms of salt tolerance in cotton. Through transcriptome analysis by RNA-Seq, we successfully identified 43,219 unigenes in *G. davidsonii.* Compared to *G. raimondii*, there were 6,173 novel genes in the *G. davidsonii* transcriptome. Among these unigenes, 4,744 and 5,337 were differentially induced by salt stress in roots and leaves, respectively. Overall, there were many more DEGs in the leaves than in the roots. During the early stages of salt stress (12 h and 24 h), the number of DEGs in roots exceeded that in leaves. However, the opposite was seen at the late stages of salt stress (Fig. 3 and Fig. S3), showing the different physiological processes in roots and leaves at distinct phases after salt treatment. DEG enrichment is very different in roots and leaves at different times of salt stress (Fig. S2). Although tissue specific DEGs occupy a prodigious proportion both in roots and leaves (61% and 65%, respectively), GO enrichment “response to stimulus” (GO:0050896) genes was most significantly enriched in leaves and roots (Fig. 5). Genes in the GO categories related to salt stress were involved in “responses to osmotic stress”, “response to oxidative stress”, “ion transport”, “response to sucrose stimulus”, as well as “response to various hormone stimulus” (Figs 6 and 7; Table S2). In addition, genes in the GO categories related to metabolic processes both in leaves and roots were involved in “hormone”, “carbohydrate”, “lipid”, “protein”, “amino”, “organic substance” and “oxidation reduction”. These results demonstrate that both roots and leaves may participate in similar pathways and molecular regulatory networks in response to salt stress.

When salt stress occurs, the stress signal is perceived by receptors and results in the generation of many secondary signal molecules, such as Ca^2+^, ROS, and hormones. This leads to the activation of related genes to induce salt stress tolerance. Of these genes, protein kinase and transcription factors act as key regulators of this process^2^. In our study, various kinds of signaling pathway-related DEGs were found (Fig. S4) and the changes in expression were consistent with previous reports. However, many unknown factors in the response to salt stress still need to be elucidated. Therefore, we particularly focused on the SOS- and ROS-related signaling pathways and photosynthesis-related metabolism.

The SOS signaling pathway plays vital roles in the maintenance of ion homeostasis. Briefly, following a Ca^2+^ spike generated in the cytoplasm after the perception of salt stress, SOS3 appeared to function as a primary calcium sensor by binding Ca^2+^ and activating SOS2. Ultimately, interactions between SOS3 and SOS2 lead to the activation of SOS1, resulting in the extrusion of Na^+^ from the cytosol^50^. However, in present study, several SOS2 and one SOS1 genes were up-regulated, while the expression of SOS3 was unchanged. More recently, SOS3-like Calcium Binding Protein 8 (SCaBP8) has been shown to be an alternative regulator of SOS2^43^. Du *et al.*^51^ and Lin *et al.*^52^ demonstrated the surmise successively in *Arabidopsis*. In line with this hypothesis, we found that several *SCaBP8* genes were up-regulated. Therefore, we speculated that *SCaBP8–SOS2–SOS1* signaling is paramount in the regulation of Na^+^ exclusion and cellular ion homeostasis in cotton. Furthermore, the SOS1 mutant was the most sensitive to salt stress, not SOS3 or SOS2 mutants^53^, suggesting that SOS1 could be regulated by other signaling pathways. Indeed, SOS1 is a target of the phospholipase D (PLD) signaling pathway in ion sensing under salt stress. Rapid and transient accumulation of phosphatidic acid (PA) results from the increased enzyme activity of PLDα1. PLDα1 activates MPK6, which can directly phosphorylate SOS1 under salt stress in *Arabidopsis*^54^. In addition, there are some cris-elements related to transcription factors such as MYB, AP2/EREBP, and TCP in the promoter region of SOS2^50^, which demonstrates that SOS2 may be regulated by several upstream transcription factors that are up-regulated during salt stress (Fig. S5), leading to the activation of SOS1. Moreover, the loss and gain-functions of SOS1 have shown that SOS1 is critical for salt tolerance but over-expression does not result in a major improvement in tolerance^55^. Therefore, additional entities must be involved in ion homeostasis. *HKT1*, which encodes a K^+^ transporter, was down-regulated at late stages after salt stress treatment in leaves, and at all stages except for 48 h in roots, likely leading to a decrease in Na^+^ and K^+^ influx. As this is a Na^+^-K^+^ co-transporter, this also suggests that Na^+^ competes with K^+^ uptake and may also block K^+^ specific transporters. Interestingly, *KUP1* in roots and *KUP2* in leaves were up-regulated, likely leading to further K^+^ influx and maintaining the K^+^ balance of the cell. However, the signaling pathways that these genes are involved in remain elusive. Together, these signaling pathways caused the lower Na^+^ content and Na^+^/K^+^ values found in the roots and leaves of *G. davidsonii* (Fig. 1b,f).

Photosynthesis plays a central role as an energy source for plant metabolism^56^. As Fig. 1 shows, photosynthesis in cotton leaves is been affected by salt stress. When suffering osmotic stress, plants will close their stomata via ABA, ROS, and MAPK cascades^7^. This simultaneously restricts the entry of CO_2_ into the leaf, reducing the rate of photosynthesis. In our study, the regulators participating in these signaling pathways were found and the gene expression was consistent with previous reports. However, in prolonged exposure to salt stress, NaCl may directly inhibit photosynthesis by inhibiting the light reaction^57^. In the present study, light reaction-related genes, including *LHC*, *PSB*, *PEI*, and *PSA*, were almost all down-regulated at 96 h after salt stress, suggesting that electron transport and the supply of NADPH for carbon fixation were limited^58^. This process was also confirmed by the reduced abundance of the large and small subunits of RuBisCO, which is a key enzyme in the first step of carbon fixation^44^,^57^. However, the down-regulation of RuBisCO caused by the reduction in CO_2_ influx or the inactivation of the light reaction needs to be further explored. In addition, proteins involved in energy metabolism were also severely affected by salt stress. ATP synthase is an important enzyme that provides energy for the cell to use through the synthesis of ATP by proton-motive forces^59^. In the present study, the abundance of eight ATP synthases was lower after exposure to salt stress, and this was consistent with previous results. In addition, when the activity of ATP synthases is inhibited, the plant is liable to suffer from oxidative stress either via the photoreduction of O_2_ to form superoxides or through the interaction of triplet-excited chlorophyll to cause singlet excited oxygen fixation^60^. Altogether, to maintain photosynthetic capacity, enhanced electron transport, reduced risk of ROS production, and improved carbon fixation will allow cotton to survive under salt stress conditions.

Absorption of sunlight leads to ROS formation, mainly in the chloroplast^61^. In response to salt stress, the generation of ROS is also achieved by the activation of ROS-producing genes, such as *RBOHs*. It has been demonstrated that ROS are produced by *RBOH* in a Ca^2+^-dependent manner^62^. Excess generation and accumulation of ROS cause damage to cellular membranes by lipid peroxidation, which is measured by MDA content (Fig. 1d,h). However, plants have evolved a series of mechanisms for ROS homeostasis. In our study, we found that most *GST* and *GRX* genes were expressed at higher levels under salt stress. The enzymes encoded by these genes play important roles in peroxide detoxification by catalyzing GSH to GSSG^63^. In addition, *POD* and CAT were found to be differentially expressed and this result was also consistent with previous reports that *GhCAT1* acts as an ROS scavenger and participates in salt stress in cotton^24^. These results suggest that GST, CAT, and POD may be the main scavengers of ROS in salt stress. Prior to their detoxification, genetic evidence suggests that ROS can also act as a signaling molecule in regulating diverse functions in plants^64^. It has been demonstrated that the *MAPK* cascade *MEKK1-MKK2-MPK4/6* could work downstream of ROS, participating in both abiotic and biotic stress signaling^16^. Additionally, *bHLH92* and *WRKY33* could participate in ROS signaling by targeting peroxidases and glutathione-S-transferases^65^. Taken together, these results show that the ROS signaling pathway plays an important role in oxidative stress by stabilizing cellular membranes. However, ROS function not individually, but synergistically with other signaling pathways, and can be regulated by transcription factors.

Alternative splicing of pre-mRNAs in higher eukaryotes became the focus of research into major sources of protein diversity in the post-genomic era^66^. However, the extent and complexity of alternative splicing in plants is not well characterized, especially for cotton. In our study, four main alternative splicing patterns were all detected (Fig. 8) and IR pattern is the most prevalent splicing pattern both in roots and leaves (Fig. S5 and Table S3). This result is consistent with the findings of other researchers in *Arabidopsis*^49^. Furthermore, alternative splicing events were significantly improved when suffering salt stress, especially for AA, AD events (Fig. S5). Indeed, alternative splicing events based on AA and AD splice sites more easily lead to functionally relevant changes in the protein products^67^. Moreover, we found parts of these alternative splicing events are tissue-specific (Fig. S5). In addition, gene annotation implied that several alternatively spliced genes were involved in abiotic stress, such as *MAPK*, *bHLH* and zinc finger transcription factors, and cytochrome *P450*. This means alternative gene splicing must play important roles in the regulation of gene expression. Taken together, these results suggest that alternative splicing may enhance plants to cope with salt stress via transcriptome plasticity^49^. However, the mechanism needs to be further explored.

All of the signaling and metabolic pathways described could regulate gene expression involved in protecting plants from salt stress at different levels, including genes encoding osmoprotectants, detoxifying enzymes, transporters, and regulatory proteins such as transcription factors, protein kinases, and phosphatases. Ultimately, these enhance salt tolerance and adaptation through ion homeostasis, osmotic homeostasis, and oxidation balance (Fig. 10). However, the response to salt stress is an all-dimensional and multitier event. We are still far from determining the full mechanisms of the response to salt stress in cotton. Even so, large numbers of key molecular factors have been used in genetic engineering to generate salt-tolerant plants, including cotton^68^. Hence, the selection of the optimum candidate genes is particularly important. An alcohol dehydrogenase1 gene identified in our study, which exhibits continuous up-regulation and co-expression in roots and leaves after salt stress (Fig. 4), could be a candidate gene for further investigation and genetic engineering; particularly since it has been demonstrated that the alcohol dehydrogenase1 gene is responsible for salt tolerance in other species^31^,^32^.

## Materials and Methods

### Plant material and salt stress conditions

Three cotton accessions, diploid wild cotton species *G. davidsonii* and two *G. hirsutum* cultivars, ZS9612 and Z9807, with sensitivities and insensitivities to salinity stress, respectively, were used for the study. Cotton seeds were surface-sterilized with 70% ethanol for 30–60 s and 10% H_2_O_2_ for 60–120 min, followed by washing with sterile water. Sterilized seeds were germinated at 26 °C under long day conditions in a 16 h light/8 h dark cycle with a light intensity of 150 μmol m^−2^ s^−1^ on 1/2 MS solid medium. Three days after germination, the plants were transferred to 1/2 Hoagland nutrient solutions at pH 6.0. For salinity stress treatment, seedlings containing two simple leaves and one heart-shaped leaf were randomly selected cultured in 1/2 Hoagland solutions supplemented with 200 mM NaCl. After exposure for 12, 24, 48, 96, and 144 h, the leaf and root samples were frozen in liquid N_2_ and stored at −70 °C for further use. Plant seedlings grown in normal 1/2 Hoagland nutrient solution was used as controls. All the cotton plants cultured in 1/2 Hoagland solutions were grown in chambers under long day conditions with a 16 h light/8 h dark cycle at 28/25 °C in Nanjing Agricultural University. The 1/2 Hoagland nutrient solution was changed every day.

### Measurement of physiological and biochemical indexes

Leaf relative water content (RWC) was measured using the method described by Barrs^69^. The total chlorophyll content of leaves was measured spectrophotometrically following the method described by Arnon^61^. Osmotic adjustment measurement includes the measurement of free proline and total soluble sugar levels. The free proline content of roots and leaves was measured spectrophotometrically according to the method described by Bates *et al.*^54^. Malondialdehyde (MDA) levels were assessed by measuring thiobarbituric acid reactive substances (TBARS)^70^. Levels of superoxide dismutase (SOD), one of the most important protective enzymes in the response to salt stress, were determined according to the protocol described by Paoletti *et al.*^71^. Concentrations of Na^+^ and K^+^ in roots and leaves were determined using a flame emission spectrophotometer at 589 nm and 767 nm, respectively. To achieve this, dry samples (0.1 g) were completely digested in 6 mL 65% HNO_3_, and 30% H_2_O_2_ was added to the reaction 5–6 times to deplete the HNO_3_. The solution was filtrated though filter paper and used for measurement.

### RNA extraction, cDNA library preparation, and RNA-Seq

Total RNA was extracted from roots and leaves by the cetyl trimethylammonium bromide (CTAB)-sour phenol extraction method^64^. The RNA was digested with RNase-Free DNase (Qiagen) and checked for integrity by capillary gel electrophoresis. Library preparation for RNA-Seq was performed using the TruSeq RNA Sample Preparation Kit (Illumina, Cat.NRS–122–2002) with 500 ng of total RNA. Accurate quantitation of cDNA libraries was performed using the QuantiFluor dsDNA System (Promega). The size range of the final cDNA libraries was determined by applying the DNA 1000 chip on the Bioanalyzer 2100 (Agilent; 280 bp). The cDNA libraries were amplified and sequenced using the cBot and HiSeq2000 systems from Illumina. Two biological replicates from each sample were used for all RNA-Seq experiments.

### Reads mapping, transcript assembly, and differential expression

After preprocessing the RNA-Seq data with an NGS QC toolkit^72^, the reads were mapped to the *G.raimondii* genome using a Tophat spliced aligner^29^. Default Tophat parameters, which allow up to two mismatches and report up to 20 alignments for reads mapping at multiple positions, were used. The sequence alignment/map files generated by Tophat were used as the input to the software Cufflinks^30^, which assembles the alignments in the sequence alignment/map file into transfrags. Cufflinks does this assembly independently of the existing gene annotations and constructs a minimum set of transcripts that best describes the RNA-Seq reads. The unit of measurement used by Cufflinks to estimate transcript abundance is FPKM. The Cufflinks statistical model probabilistically assigns reads to the assembled isoforms. Cuffmerge was used to merge these four assemblies with the reference annotation (*G.raimondii*_221_v2.1.gene.gff) into a single gtf file that was used later to identify differentially expressed genes. The class codes in the Cuffmerge output were used to identify novel isoforms, intergenic transcripts, and splice junctions. Lastly, Cuffdiff was used to find DEGs. A *q* value cutoff of 0.05 was used to determine whether a gene had differential expression between two biological repeats. Additionally, one of the two tissues was required to have RPKM >1. Using an empirical method^73^, 2.3 FPKM was chosen as the expression cutoff for alternative splicing isoforms. In addition, the AS isoforms that were identified in both replications, were regarded as the stable isoforms. We used the ASTALAVISTA software^74^ to quantify the type of AS events based on the assembled transcripts by the Cufflinks software.

### Validation of RNA-Seq data by real time RT-PCR

To verify the differential expression detected by the Illumina RNA-Seq data, real-time RT-PCR (qRT-PCR) was performed on a new set of 3 replicates for each sample. A set of 30 genes was chosen randomly (Table S6), including 10 up-regulated, 10 unchanged, and 10 down-regulated genes from roots and leaves by dividing their expression level at different time points with their observed RPKM. qRT-PCR was performed using a Bio-Rad CFX96 Real-Time instrument and the light cycler fast start DNA Master SYBR Green I kit (Roche, Basel, Switzerland). Reactions were performed in triplicate, and contained 100 ng of cDNA, 0.5 μL of each primer (10 μM/μL), and 10 μL SYBR Green Master Mix in a final volume of 20 μL. The amplification reactions were performed under the following conditions: 95 °C for 5 min, followed by 40 cycles of 95 °C for 15 s, 58 °C for 20 s, and 72 °C for 30 s. Melting curve analysis, performed by increasing the temperature from 55 °C to 95 °C (0.5 °C per 10 s), and gel electrophoresis of the final product confirmed the presence of single amplicons. Relative fold differences for each sample in each experiment were calculated using the ΔΔCt method^75^. The *GhHis3* gene was used as a control. To corroborate the expression levels measured by RNA-Seq, the ratio of expression levels between tissues using RNA-Seq was compared to the ratio of expression as measured by qRT-PCR. In addition, RT-PCR and qRT-PCR were used to validate the alternative splicing of five types found in roots or leaves by RNA-Seq (Table S7).

### Go enrichment and pathway analysis

AgriGO software^35^ was used for gene ontology analysis, and Singular Enrichment Analysis (SEA) was performed. The input sample list was the *G. raimondii* gene ID, which was converted from the original ID of the Cuffdiff default configuration, and the background was all the annotated genes in *G. raimondii*. The output of enrichment needed FDR < 0.05. The MapMan tool facilitates the classification of transcripts into hierarchical categories (known as bins) in a manner that alleviates the redundancy present in other commonly used ontologies^76^; therefore, the tool provides an additional level of analysis beyond the functional enrichment of typical GO categories. Using this schema, the user may view a metabolic pathway or process of interest annotated by groups of participatory entities.

### Data Section

RNA-Seq data in this study have been deposited at the NCBI under the accessions SRP061663.

## Additional Information

**How to cite this article**: Zhang, F. *et al.* Genetic regulation of salt stress tolerance revealed by RNA-Seq in cotton diploid wild species, *Gossypium davidsonii*. *Sci. Rep.* **6**, 20582; doi: 10.1038/srep20582 (2016).

## Supplementary Material

Supplementary Information

## Figures and Tables

**Figure 1:** Physiological analysis of *G. davidsonii* and *G. hirsutum* in response to various durations of salt stress. (**A**) Phenotype of *G. davidsonii* and *G. hirsutum* cv. ZS9612 at 144 h post salt stress (200 mM NaCl). (**B**) Various physiological index involved in salt stress on roots and leaves indicated. (**a**) Leaf photosynthetic rate (Pn) fold changes at different times post salt stress. (**b**–**e**) Leaf Na^+^/K^+^ ratio, SOD, MDA, and proline fold changes at different time post salt stress. (**f**–**i**) Root Na^+^/K^+^ ratio, SOD, MDA, and Proline fold changes at different times post salt stress. *G. davidsonii* seedlings grown under normal conditions were used as controls. At least three biological replicates were used. Multiple comparisons were performed with significant difference in different letter at P < 0.05 level; Error bars represent SD.

**Figure 2:** Workflow of RNA-Seq analysis. (**A**) Clean data sets were generated from 40 samples with two independent biological replicates of roots and leaves at five time points. (**B**) The reads were mapped using Tophat onto the *G. raimondii* genome. (**C**) Cufflinks was used for transcriptome reconstruction, resulting in 40 different assemblies corresponding to 40 samples. (**D**) Cuffmerge was used to merge the four assemblies and the reference annotations into a single consensus list of transcripts and to categorize the assembled transcripts. (**E**) Cuffdiff was used to identify differentially expressed genes (DEGs) under salt stress in both tissues at five time points. (**F**) AgriGo was used to identify enriched GO terms. (**G**) Mapman was used to enrich DEGs in the pathway related to salt stress.

**Figure 3:** Analysis of global differential expressed genes. (**A**) DEGs in roots and leaves under salt stress. (**B**) Number of DEGs in each of the samples at five time points. (**C**) Venn diagram of the 4,744 DEGs in roots. (**D**) Venn diagram of the 5,337 DEGs in leaves.

**Figure 4:** Heat map of DEGs at five time points in roots and leaves. (**A**) Heat map depicting log_2_^(fold change)^ of common differentially expressed genes in roots; (**B**) Heat map depicting log_2_^(fold change)^ of common differentially expressed genes in leaves. Red and green colors indicate up- and down- regulated transcripts, respectively, from both control and salt treated tissues. False Discovery Rate (FDR) ≤ 0.001 and the maximum value of |log2 (ratio of stress/control)| ≥ 1 was used as the cut-off to evaluate significant differences in expression). Red arrow: Alcohol dehydrogenase (ADH) in roots and leaves, respectively; Black arrow: UDP-Glycosyltransferase in roots and leaves, respectively.

**Figure 5:** GO category of all DEGs at the second level in roots and leaves. The size of blue block in the outer loop indicates the DEG numbers in each GO term. The color of the outer blue loop indicates the FDR value of the GO term: a deeper color represents a smaller FDR value. The pink range indicates signification enrichment, with FDR ≤0.05 as the cutoff. (**A**) GO category of DEGs in roots. (**B**) GO category of DEGs in leaves.

**Figure 6:** Agri GO analysis of DEGs in roots. Singular enrichment analysis was performed in AgriGO to identify enriched gene ontologies associated with high tillering lines. Each box shows the GO term number, the p-value in parenthesis, and GO term. The pair of numerals in the left represents number of genes in input list associated with that GO term and number of genes in input list. The pair of numerals in the right represents number of genes associated with a particular GO term in the *Gossypium* database and total number of *Gossypium* genes with GO annotations in the *Gossypium* database. Box colors indicate levels of statistical significance: yellow = 0.05; orange = e^−5^; and red = e^−9^.

**Figure 7:** Agri GO analysis of DEGs in leaves. Statistical standards are as in Fig. 6.

**Figure 8:** Validation of alternative splicing detected by RNA-Seq through RT-PCR and qRT-PCR. (**A**) Models for different alternative splicing patterns. Black boxes indicated exons, thick solid lines indicated introns, and flexed lines indicated splice junctions. (**B–F**) Validation of selected genes with IR (12 h), AA (24 h), ES (48 h), MEE (96 h) and AD (144 h) splicing detected by RNA-Seq analysis both in roots and leaves of *G. davidsonii*. CK, cotton plants grown under normal conditions; Salt: cotton plants grown under 200 mM NaCl. At least three biological replicates were used. “*” means significant difference at P < 0.05 level; “**” means significant difference at P < 0.01 level. Error bars represent SD.

**Figure 9:** qRT-PCR validation of transcript levels evaluated by RNA-Seq in roots and leaves of *G. davidsonii* under 200 mM NaCl stress conditions. (**A,B**) represent the correlation of the fold change analyzed by RNA-Seq platform (x-axis) with data obtained using real time PCR (y-axis) in roots and leaves of *G. davidsonii*. 30 independent genes were randomly selected: 10 up-regulated genes, 10 unchanged genes and 10 down-regulated genes. Three biological replicates were used from each sample at five time points post salt stress.

**Figure 10:** Model of the complex regulatory networks activated in response to salt stress in cotton. Salt stress is first sensed by an unidentified mechanism. A Ca^2+^ spike generated in the cytoplasm activates the ROS (black route) and SOS (green route) pathways. In addition, photosynthetic pathways and metabolism in leaves (green boxes) were found to be changed to allow plants to adapt to osmotic and ionic stress at 96 h after salt stress. Meanwhile, other signaling methods such as hormones, and CDPK signaling factors, together alter the global transcriptional profile, resulting in gene expression and the activation of cellular detoxification mechanisms for ion homeostasis, osmotic homeostasis, and redox balance in plants. Transcription factors that were found to play important roles in SOS and ROS pathways are not displayed this figure. R12-R144 h and L12-L144 h indicate the different time points after salt stress in roots and leaves, respectively. Bar, log_2_ (fold change of DEGs).

**Table 1:** Numbers of transcripts and unigenes assembled by Cufflinks.

Class	Total transcript	Total gene	Novel gene	Annotation gene
RC	112144	39861	2864	36997
RS	118405	40916	4179	36737
LC	117358	42232	5230	37002
LS	117003	40942	3952	36990
total	157953	43219	6245	37046

RC: root well-watered control; RS: root salt-stressed treatment; LC: leaf well-watered control; LS: leaf salt-stressed treatment.
